The article "Study on the Efficacy and Safety of Oral Care in ICU Patients Based on Meta-Analysis" was retracted in 2023. Reasons: signs of a paper mill; suspected computer-generated content; unreliable results or conclusions; concerns about the data.

# Study on the Efficacy and Safety of Oral Care in ICU Patients Based on Meta-Analysis

**DOI:** 10.1155/2022/5337181

**Published:** 2022-10-07

**Authors:** Yang Gao, Huifen Xu, Yahui Yang, Juan Wu

**Affiliations:** ^1^Department of Critical Care, Affiliated Hospital of Nantong University, Nantong 226001, China; ^2^NantongUniversity, Nantong 226019, China; ^3^Department of CCU, Affiliated Hospital of Nantong University, Nantong 226001, China

## Abstract

The effectiveness and safety of oral care in Intensive Care Unit (ICU) patients by meta-analysis are explored. According to the research direction of the effectiveness and safety of oral nursing in ICU patients, the corresponding literature studies are retrieved in literature databases and meta-analysis is performed. A total of 17 Chinese and English literature studies are included, and the literature has no obvious publication bias. The experimental results show that the improvement effect of dry mouth and halitosis in the improved group is significantly higher than that in the traditional group, and the dry mouth score, plaque index, and complications such as oral mucosa infection, oral mucosa damage, and halitosis are significantly reduced in the improved group, and the differences are statistically significant (*P* < 0.05). Improved oral care can significantly improve the symptoms of dry mouth and halitosis in ICU patients, quickly remove dental plaque and effectively reduce the incidence of complications such as halitosis, oral mucosal infection, and oral mucosal damage. Improved oral care is an effective and safe ICU nursing program.

## 1. Introduction

The condition of patients in Intensive Care Unit (ICU) is in crisis, and most ICU patients will have uncomfortable symptoms such as dry mouth and thirst. At present, effective clinical intervention guidelines for dry mouth and thirst in ICU patients have not been explored, resulting in increased difficulty of disease treatment for patients. It has adverse effects on the smooth progress of diagnosis and treatment of patients and the improvement of prognosis [1]. Previous studies have pointed out that the combined application of artificial saliva, lemon juice and other alternative products in the process of oral care can effectively improve the symptoms of dry mouth, and cold water stimulation is also a new intervention program to reduce the degree of dry mouth, and has achieved certain effects in the improvement of dry mouth symptoms [2, 3].

Existing literature on ICU patients with oral cavity nursing intervention is applied to the clinical curative effect and safety of literature is relatively more, but the data is relatively fragmented and has not been unified analysis summary. Therefore, this paper used meta-analysis to further explore the clinical efficacy and application safety of oral nursing intervention in improving dry mouth symptoms in ICU patients. It can provide a new idea for the oral care management of ICU patients and the improvement of dry mouth symptoms.

The article "Study on the Efficacy and Safety of Oral Care in ICU Patients Based on Meta-Analysis" was retracted in 2023. Reasons: signs of a paper mill; suspected computer-generated content; unreliable results or conclusions; concerns about the data.

The rest of this paper is organized as follows: Section 2 discusses related work, followed by literature information and statistical methods designed in Section 3.  Section 4 shows the experimental results and analysis, and Section 5 is the conclusion, which briefly summarizes all of standpoints.

## 2. Related Work

When the symptoms of ICU patients with dry mouth symptoms occur, the reason is more complicated. The ICU patients are prone to electrolyte disorder, and massive blood loss during operation, the endocrine disorder, as well as the important organ failure and so on all can cause loss of body fluids and blood volume is insufficient, which can lead to high permeability and low blood volume symptoms of dry mouth. Dry mouth symptoms can reduce the patient's comfort. It will also cause anxiety and other stress emotions, further increase the oxygen consumption and metabolic burden of patients, and hinder the disease outcome and rehabilitation of patients [4].

Traditional oral care schemes such as dipping cotton swabs into moistened lips and lips have shortcomings such as fast water evaporation, poor relief effect of dry mouth, and nursing risks such as cotton wool shedding blocking esophageal airway and contusing esophageal airway and oral mucosa [5]. The results of this study first showed that the improvement effect of dry mouth symptoms and the score of dry mouth degree of patients in the improved group were significantly better than those in the traditional group, which further indicated that the implementation of a series of oral management guidance for ICU patients with the modified oral care program was helpful to promote the improvement of dry mouth symptoms of patients. The main reason may be that cold water can stimulate the brain by sensory afferent fibers surface sensory cortex, raise the excitement and inhibition of thirst reflex of the brain, at the same time, cold water stimulation can inhibit the secretion of vasopressin process to alleviate symptoms of dry mouth. The scheme has the advantage of patients and will not cause additional burden of liquid water. The application of mint, honeysuckle, and other self-made oral cleaning liquid can play a certain antibacterial effect, quickly remove oral bacteria, and maintain oral health under the condition of alleviating patients' symptoms of thirst and dry mouth through cold stimulation [6].

The article "Study on the Efficacy and Safety of Oral Care in ICU Patients Based on Meta-Analysis" was retracted in 2023. Reasons: signs of a paper mill; suspected computer-generated content; unreliable results or conclusions; concerns about the data.

The results of this study showed that by improving oral care intervention and reducing the incidence of halitosis, the application of plaque removal effect is more significant. This indicates that the use of self-made oral care solution for cleaning in the process of improving oral care and reasonable planning of oral care can quickly remove dental plaque in the mouth and avoid oral odor. The main reason was that the traditional oral care measures can remove plaque disease, eliminate halitosis, but there are still poor antibacterial effect, prevention of infection, and short oral odor retention time. Literature showed that oral care solutions made of traditional Chinese medicine can be used for oral cleaning. The active ingredients in traditional Chinese medicine such as honeysuckle, mint, and ethanol extract can play obvious anti-inflammatory, antibacterial, and bacteriostatic effects. They can effectively remove dental plaque and improve the bad breath caused by dental plaque through antioxidant and immune regulation [7].

The vast majority of ICU patients with severe illness have greatly reduced immunity, which increases inflammation in the body. The oral cavity is the main channel of the body's respiratory and digestive systems. The decreased immunity of the body leads to the increased risk of complications such as oral erosion, ulcer, and infection, which can cause local and systemic organ infections in severe cases, posing a serious threat to the health and disease treatment of ICU patients [8]. The experimental results show that the application of improved oral care intervention program can effectively reduce the risk of oral complications, which is consistent with the results of previous studies. The reason may be that patients in the ICU cannot eat normally due to the disease, and the amount of saliva in the mouth decreases, resulting in dry mouth and indirectly promoting bacterial growth, which eventually leads to oral ulcer, chyme, bacterial inflammation and other oral diseases. So the process of improving oral care can be through cold water stimulation intervention and regular cleaning teeth. Mouthwash can kill bacteria in the mouth, and at the same time, it can wash away necrotic tissues and food residues in the mouth and destroy the plant environment increased by bacteria, which can inhibit the excessive proliferation and inflammation of bacteria, and effectively reduce the risk of oral infection, erosion, ulcer and other complications [9].

## 3. Literature Information and Statistical Methods

### 3.1. Literature Search

According to the research direction of the effectiveness and safety of oral care in ICU patients, controlled clinical literature published from 2010 to 2022 are searched in the literature database. The search keywords are oral care and intensive care unit. These problems include efficacy, complications, degree of dry mouth, dental plaque index, oral mucosal infection, oral mucosal damage, halitosis, oral care, intensive care unit, plaque index, OralDiskinfection, OralDisk7 damage, and bad breath which are analyzed based on the selected literature. All the included literature carried out oral nursing intervention according to the improved nursing and traditional nursing plan, and there is no obvious loss of data. No discrimination conditions such as gender, age, nationality, and race are set in the selection of subjects in the literature, and there is no obvious loss of data. All studies are approved by medical institutions. The literature included any one or more of the outcome indicators as below: efficacy, complications, degree of dry mouth, dental plaque index, oral mucosa infection, oral mucosa damage, and halitosis. To be included in the literature, it is necessary to exclude multiple results with illogical duplication, serious missing data, obvious errors in research operation, basic experiments and other research directions or types of literature.

The article "Study on the Efficacy and Safety of Oral Care in ICU Patients Based on Meta-Analysis" was retracted in 2023. Reasons: signs of a paper mill; suspected computer-generated content; unreliable results or conclusions; concerns about the data.

### 3.2. Literature Quality Assessment

The modified Jadad scale is used to evaluate the quality of the selected literature. The total score is 1–7, ≤3 is considered as low quality literature, and vice versa is considered high quality literature.

### 3.3. Statistical Methods

RevMan5.2 statistical software is used to analyze the study data. The *RR* is used to represent the count data, the SMD is used to represent the analysis statistics, and the effect size is expressed as 95% CI. When the heterogeneity of each study meet *P* < 0.1 and *I*^2^ ≥ 50%, it is statistically significant, and the random effect model is used. Otherwise, the fixed effect model is selected. Clinical and methodological heterogeneity is analyzed descriptively.

## 4. Experimental Results

### 4.1. Characteristics of Literature Information

A total of 17 literature studies are included, with 15 Chinese and 2 English literature respectively. Among them, 6 articles are of low quality and 11 articles are of high quality. The basic information and quality characteristics of the included articles are shown in Table 1. In Table 1, ① indicates that the symptoms of dry mouth and halitosis are improved; ② indicates dry mouth score; ③ indicates plaque index; ④ indicates incidence of oral mucosal infection; ⑤ indicates incidence of oral mucosal damage; ⑥ indicates incidence of halitosis.  Figure 1 shows the flowchart of literature screening.

The article "Study on the Efficacy and Safety of Oral Care in ICU Patients Based on Meta-Analysis" was retracted in 2023. Reasons: signs of a paper mill; suspected computer-generated content; unreliable results or conclusions; concerns about the data.

### 4.2. Meta-Analysis of Literature Bias

Figure 2 shows the overall literature bias.  Figure 3 shows the bias of a single document. It can be seen from Figures 2 and 3 that there is no obvious publication bias between the 17 included Chinese and English literature studies.

### 4.3. Meta-Analysis on the Improvement of Dry Mouth and Halitosis

Five literature studies related to the improvement of symptoms of dry mouth and halitosis are included with heterogeneity (*I*^2^ > 50.00%).  Figure 4 shows the forest map of meta-analysis on the improvement of dry mouth and halitosis. It can be seen from Figure 4 that the improved nursing group significantly increases the improvement effect of oral dry mouth and halitosis (*P* < 0.00001). It is suggested that improved oral care can significantly improve the symptoms of dry mouth and halitosis in ICU patients.

### 4.4. Meta-Analysis of Differences in Dry Mouth Score

Three literature studies related to dry mouth score are included with heterogeneity (*I*^2^ > 50.00%).  Figure 5 shows the forest map of dry mouth score meta-analysis. It can be seen from Figure 5 that the dry mouth score of the modified nursing group is significantly lower and statistically different (*P* < 0.00001). It is suggested that improved oral care can significantly reduce the symptoms of dry mouth in ICU patients.

### 4.5. Meta-Analysis of Differences in Dental Plaque Index

Three literature studies related to dental plaque index are included with heterogeneity (*I*^2^ *>* 50.00%).  Figure 6 shows the forest map of dental plaque index meta-analysis. It can be seen from Figure 6 that the dental plaque index of the modified nursing group is significantly reduced and statistically different (*P* < 0.00001). It is suggested that improved oral care can significantly reduce the dental plaque index of ICU patients.

### 4.6. Meta-Analysis of Differences in Complication Rates

#### 4.6.1. Meta-Analysis of Differences in Incidence of Oral Mucosal Infections

Seven literature related to the incidence of oral mucosal infection are included (*I*^2^ < 50.00%).  Figure 7 shows the forest plot of meta-analysis on incidence of oral mucosal infection. It can be seen from Figure 7 that the incidence of oral mucosal infection in the modified nursing group is significantly lower and statistically different (*P* > 0.00001). It is suggested that the improved oral care can significantly reduce the incidence of oral mucosal infection in ICU patients.

#### 4.6.2. Meta-Analysis of Differences in the Incidence of Oral Mucosal Damage

Seven literature studies related to the incidence of oral mucosal damage are included and homogeneity is found (*I*^2^ < 50.00%).  Figure 8 shows the forest map of meta-analysis on the incidence of oral mucosal damage. It can be seen from Figure 8 that the incidence of oral mucosal damage in the modified nursing group is significantly lower and statistically different (*P* < 0.00001). It is suggested that improved oral care can significantly reduce the incidence of oral mucosal damage in ICU patients.

The article "Study on the Efficacy and Safety of Oral Care in ICU Patients Based on Meta-Analysis" was retracted in 2023. Reasons: signs of a paper mill; suspected computer-generated content; unreliable results or conclusions; concerns about the data.

#### 4.6.3. Meta-Analysis of Differences in the Incidence of Halitosis

Eight literature studies related to the incidence of halitosis are included with heterogeneity (*I*^2^ < 50.00%).  Figure 9 shows the forest map of the incidence of halitosis meta-analysis. It can be seen from Figure 9 that the incidence of halitosis in the modified nursing group is significantly lower and statistically different (*P* < 0.00001). It is suggested that improved oral care can significantly reduce the incidence of halitosis in ICU patients.

## 5. Conclusion

The application of the improved oral care solution in ICU patients can significantly improve the symptoms of dry mouth and halitosis, reduce the degree of dry mouth in patients, quickly remove plaque and improve halitosis. At the same time, the application of this program has the advantages of low incidence of complications such as infection of oral mucosa and injury of oral mucosa. Improved oral care is an effective and safe nursing plan in ICU, which is worthy of popularization and application in ICU patients.

The outcome indicators of this study are incomplete, the types of ICU diseases and the improved nursing plan are not classified in detail, and the number of included literature is relatively small. All these problems may increase the research bias of the overall data, and these shortcomings will be further optimized in the next study.

## Figures and Tables

**Figure 1:** Flowchart of literature screening.

**Figure 2:** Overall literature bias.

**Figure 3:** Bias of a single document.

**Figure 4:** Forest map of meta-analysis on the improvement of dry mouth and halitosis.

**Figure 5:** Forest map of dry mouth score meta-analysis.

**Figure 6:** Forest map of dental plaque index meta-analysis.

**Figure 7:** Forest plot of meta-analysis on incidence of oral mucosal infection.

**Figure 8:** Forest map of meta-analysis on the incidence of oral mucosal damage.

**Figure 9:** Forest map of the incidence of halitosis meta-analysis.

**Table 1:** Features of literature information.

The author	Published time	Sample size	Outcome indicators	Quality of the literature
Jin [10]	2016	45/45	①	3
Qin [11]	2015	78/78	①	3
Li [12]	2014	80/80	①	3
Chen et al. [13]	2019	30/30	①④⑤	5
Wang et al. [14]	2018	48/48	①④⑥	5
Lv et al. [15]	2021	127/125	②	4
Gu et al. [16]	2019	21/21	②	4
VonStein et al. [17]	2019	62/41	②	4
Gong et al. [18]	2018	40/40	③	4
Shu et al. [19]	2018	51/49	③④	4
Liang and Zhao [20]	2020	83/82	③④⑤⑥	5
Du et al. [21]	2017	60/60	④⑤⑥	4
Wang et al. [22]	2019	26/26	④⑥	3
Hao [23]	2013	30/30	④⑤⑥	4
Kou [24]	2011	100/100	⑤⑥	3
Zhang et al. [25]	2011	100/100	⑤⑥	3
Zhou [26]	2019	635/635	⑤⑥	4

The article "Study on the Efficacy and Safety of Oral Care in ICU Patients Based on Meta-Analysis" was retracted in 2023. Reasons: signs of a paper mill; suspected computer-generated content; unreliable results or conclusions; concerns about the data.

## Data Availability

The simulation experiment data used to support the findings of this study are available from the corresponding author upon request.
